# Protein tyrosine phosphatase Meg2 dephosphorylates signal transducer and activator of transcription 3 and suppresses tumor growth in breast cancer

**DOI:** 10.1186/bcr3134

**Published:** 2012-03-06

**Authors:** Fuqin Su, Fangli Ren, Yu Rong, Yangmeng Wang, Yongtao Geng, Yinyin Wang, Mengyao Feng, Yanfang Ju, Yi Li, Zhizhuang J Zhao, Kun Meng, Zhijie Chang

**Affiliations:** 1 State Key Laboratory of Biomembrane and Membrane Biotechnology, School of Medicine, School of Life Sciences, Tsinghua University, Beijing 100084, China; 2 Department of Pharmacology, Qiqihar Medical Collage, Qiqihar 161006, China; 3 Department of Oncology, Chinese PLA General Hospital, Beijing 100853, China; 4 School of Life Sciences, Peking University, Beijing 100080, China; 5 Department of Pathology, University of Oklahoma Heath Science Center, Oklahoma City, Oklahoma 73104. USA; 6 Beijing Cell Technology Inc., Beijing 100080, China

## Abstract

**Introduction:**

Signal transducer and activator of transcription 3 (STAT3) is over-activated or phosphorylated in breast cancers. The hyper-phosphorylation of STAT3 was attributed to either up-regulated phosphorylation by several tyrosine-kinases or down-regulated activity of phosphatases. Although several factors have been identified to phosphorylate STAT3, it remains unclear how STAT3 is dephosphorylated by PTPMeg2. The aim of this study was to determine the role of PTPMeg2 as a phosphatase in regulation of the activity of STAT3 in breast cancers.

**Methods:**

Immunoprecipitation assays were used to study the interaction of STAT3 with PTPMeg2. A series of biochemistry experiments were performed to evaluate the role of PTPMeg2 in the dephosphorylation of STAT3. Two breast cancer cell lines MCF7 (PTPMeg2 was depleted as it was endogenously high) and MDA-MB-231 (PTPMeg2 was overexpressed as it was endogenously low) were used to compare the level of phosphorylated STAT3 and the tumor growth ability in vitro and in vivo. Samples from breast carcinoma (n = 73) were subjected to a pair-wise Pearson correlation analysis for the correlation of levels of PTPMeg2 and phosphorylated STAT3.

**Results:**

PTPMeg2 directly interacts with STAT3 and mediates its dephosphorylation in the cytoplasm. Over-expression of PTPMeg2 decreased tyrosine phosphorylation of STAT3 while depletion of PTPMeg2 increased its phosphorylation. The decreased tyrosine phosphorylation of STAT3 is coupled with suppression of STAT3 transcriptional activity and reduced tumor growth *in vitro *and *in vivo*. Levels of PTPMeg2 and phosphorylated STAT3 were inversely correlated in breast cancer tissues (P = 0.004).

**Conclusions:**

PTPMeg2 is an important phosphatase for the dephosphorylation of STAT3 and plays a critical role in breast cancer development.

## Introduction

STAT3 is crucial in regulating cell growth, differentiation and survival in response to many extracellular cytokines and growth factors [1,2]. Hyper-phosphorylation of STAT3 has been observed in a variety of hematopoietic malignancies and solid tumors, including breast cancer [3,4]. In general, latent cytoplasmic STAT3 becomes activated through phosphorylation at the residue Tyr705 by Janus Associated Kinase (JAK) or growth factor receptor-associated tyrosine kinase (Src). Phosphorylated STAT3 dimerizes through a reciprocal Src homology 2-phospho-tyrosine interaction and accumulates in the nucleus, where it activates the transcription of a wide array of genes, including Bcl-xl, cyclin D1, c-Myc and SOCS3 [5].

Most studies attributed the hyper-phosphorylation of STAT3 to over-activation of JAK or Src kinase. However, STAT3 phosphorylation is also tightly regulated by a process of dephosphorylation, which is mediated by protein tyrosine phosphatases (PTPs). A line of evidence has been provided that phosphatases play an important role in numerous signaling pathways that regulate cell proliferation, apoptosis, adhesion, and migration [6]. PTPs are a large and structurally diverse family of enzymes that catalyze the dephosphorylation of phosphorylated proteins. Previous studies indicated that protein tyrosine phosphatase 1B (PTP1B) modulates cytokine signaling pathways by dephosphorylating JAK2, TYK2, STAT5a/b [7,8], and STAT6 [9] in the nucleus. Other studies demonstrated that STAT1, STAT3 and STAT5 are dephosphorylated by SHP2 [10-12] and TC-PTP (PTPN2) [13,14] in the nucleus. It appears that STAT proteins can be dephosphorylated by different phosphatases both in the cytoplasm and nucleus [15]. Importantly, aberrant expression of PTPs leads to hyper-phosphorylation of STATs in the development of human diseases, including cancers, diabetes, inflammation and infectious diseases [16,17].

PTPMeg2 (PTPN9, protein tyrosine phosphatase, non-receptor type 9), a cytoplasmic phosphatase cloned with sequence homology to retinaldehyde-binding protein and yeast SEC14p, is reported to dephosphorylate EGFR, ErB2 and Fox-1 [18-20]. Functional studies indicated that PTPMeg2 promotes intracellular secretary homotypic vesicle fusion in hematopoietic cells [21], regulates embryonic development [22] and controls expansion of erythroid cells [23]. Other studies demonstrated that PTPMeg2 regulates insulin production, beta cell growth or insulin signaling by reducing insulin receptor dephosphorylation in type II diabetes [18,19]. Recently, two studies showed that PTPMeg2 promotes dephosphorylation of EGFR and ErbB2 thereafter to impair the activation of STAT3 [20] and STAT5 [20,24] in breast cancer cells. However, it remains unknown whether PTPMeg2 directly targets STAT3. In this study, we demonstrated that PTPMeg2 dephosphorylates STAT3 at the Tyr705 residue by a direct interaction. We propose that PTPMeg2 is a novel direct phosphatase for STAT3.

## Materials and methods

### Cell culture, reagents and plasmid construction

MCF7, MDA-MB-231, and HEK293T cells were obtained and characterized by a cytogenetic analysis by American Type Culture Collection (ATCC) and maintained in this lab according to the recommendation of ATCC. The cell lines were characterized in this lab by morphological analysis before using for experiments. The v-Src/NIH3T3 cell line was a gift from Dr. H Yu at City of Hope Comprehensive Cancer Center, California, USA and was characterized by morphological analysis in this lab according to her recommendation. The stable cell line for depletion of PTPMeg2 by shRNA was generated in this lab based on MCF7 and characterized by morphological analysis and the expression of targeted gene was characterized by a Western blot. The cells were cultured in DMEM medium supplemented with 10% fetal bovine serum in 5% CO_2 _astrosphere in 37°C. The mouse hepatic cell lines STAT3^-/- ^(KO) and STAT3^+/+ ^(WT) derived from STAT3 conditional knockout and wild-type mice were also cultured in DMEM medium.

Anti-sera against PTPMeg2 were generated by immunizing rabbits with purified GST-PTPMeg2 (1-1779) proteins in ZJ Zhao's lab. Anti-Myc (9E10), anti-HA (F-7), anti-GFP (FL), anti-pSTAT3(Tyr705, B-7), anti-pSTAT3(Ser727), anti-STAT3 (F-2) and anti-STAT3 (C-20) antibodies, and protein G/A plus agarose beads were purchased from Santa Cruz Biotechnology, and anti-β-Actin (AC-15) antibody from Sigma. MG132 and leupepstin were purchased from Amresco (AMRESCO Inc. OH), and human recombinant IL-6 and IL-6 receptor from B&D (B&D SYSTEM, USA). Plasmids including GST-STAT3, pXJ40-STAT3, and its deletions were kindly provided by Dr. Xinmin Cao [25]. Expression vectors for human PTPMeg2 and PTPMeg2C515S or deletion mutants were constructed based on pcDNA3.1-Myc or pEFneo-Myc. Other plasmids involved in this study were stored in the lab.

### Luciferase assay

MCF7 cells were plated in 24-well plates the day before transfection. An amount of 0.1 μg of reporter plasmid pAPRE-luc or M67-luc together with 5 ng of an internal control plasmid pRL-TK was transfected. Constructs expressing STAT3, PTPMeg2 and its mutants were co-transfected at an amount of 0.4 μg per well. To deplete endogenous PTPMeg2, 0.8 μg of vectors with shRNA targeting PTPMeg2 (shRNA1: 5'-GATCCGGAAAGGCATTGTAAATTCAAGAGATTTACAATGCCTTCCTTCCTTA-3', shRNA2: 5'-GATCCGCAAGGAATCTATGAGGAATTCAAGAGATT CCTCATAGATTCCTTGCTTA-3', shRNA3: 5'-GATCCCTAGAGTGAAGCT AACAATTCAAGAGATTGTTAGCTTCACTCTAGTTTA-3') in pSilencer-4.1 was transfected. Twenty-four hours after transfection, luciferase assays were performed with a dual-luciferase reporter assay system (Vigofect Inc. Beijing, China) and the luciferase activity was normalized by firefly against the renilla luciferase activity.

### Western blot, GST pull down and immunoprecipitation assay

Proteins were analyzed by SDS-PAGE and Western blot [26]. For immunoprecipitation experiments, HEK293T cells grown in 60 mm dishes were transfected with indicated expression plasmids and were lysed in cell lysis buffer (20 mM Tris-Cl, pH 7.6, 150 mM NaCl, 5 mM EDTA, 10 mM MgCl_2_, 0.5% NP40, 10% glycerol, 1 mM DTT, 0.1 mM Na_3_VO_4_, 1 mM phenylmethylsulfonyl fluoride, 1 μg/ml aprotinin, 1 μg/ml leupeptin, and 1 μg/ml pepstatin) for 30 min on ice, and then the lysates were centrifuged at a maximum speed for 15 min. Supernatants of cell lysates were incubated with 2 μg of indicated antibodies overnight at 4°C, and 30 μl of protein IgG/A agarose plus beads were added for binding for 4 h at 4°C. Beads were washed with cell lysis buffer (containing 0.1 mM vanadium) 4 times and bound proteins were eluted with 2 × loading sample buffer and analyzed by Western blot with indicated antibodies. For GST-pull down assays, the procedure was similar to that in immunoprecipitation experiments except that GST beads were used and washed by PBST buffer.

### In vitro dephosphorylation assay

GST-PTPMeg2 WT and GST-PTPMeg2CS proteins were expressed and purified as described previously [27]. Phosphorylated Flag-STAT3 was prepared from HEK 293T cells transfected with Flag-STAT3 for 48 h and then stimulated with IL-6 for 30 min. Purified phosphorylated Flag-STAT3 was incubated with GST and GST-PTPMeg2 WT or GST-PTPMeg2CS proteins at 37°C for 30 min with PTPase reaction buffer (25 mM Tris-Cl, pH 7.5, 2.5 mM EDTA, 1 mM EGTA, 1 mg/ml BSA, 10 μM TPCK, 1 mM Benzamidine, 5 mM DTT, 1 mM phenylmethylsulfonyl fluoride, 1 μg/ml aprotinin, 1 μg/ml leupeptin, and 1 μg/ml pepstatin). The dephosphorylation reaction was terminated by directly boiling. Proteins were separated with SDS-PAGE and analyzed with an anti-pSTAT3 and anti-Flag antibodies by a Western blot.

### Immunocytochemistry

Cells were seeded on glass coverslips for 24 h and subjected to serum-starvation for 18 h before treatments with IL-6 for 30 min. Cell was fixed in 4% paraformaldehyde for 20 min at 4°C and permeabilized in 0.3% Triton X-100 for 15 min. Cells were blocked with 10% normal rabbit serum at room temperature and incubated in primary antibody overnight at 4°C. Primary antibodies used were an anti-PTPMeg2 or an anti-Flag antibody. Secondary antibodies used were FITC-conjugated and TRITC-conjugated IgG. Nucleus was stained with DAPI.

### Cell growth experiment

MCF7 cells stably transfected with the shPTPMeg2 plasmid, or MDA-MB-231 or mouse hepatic STAT3 KO cells infected with an adenovirus for over-expression of PTPMeg2, were seeded on 96-well plates at a density of 1000 cells/well in triplicate. Cells were cultured for different times and 5 g/L of MTT was added 4 h before termination of cell growth. The purple blue sediment was dissolved in 150 μl of DMSO before harvest. The relative optical density (OD)/well was determined at wavelength of 570 nm in a WELLSCAN MK3 ELIASA (Lab systems, Dragon, Finland) using a 630 nm reference filter. Cell growth curve was drawn according to the average of OD570-OD630.

### Xenograft tumor model

Exponentially growing MCF7 cells were stably transfected with the PTPMeg2 shRNA vector and MDA-MB-231 were infected with the adenovirus or retrovirus and v-Src/NIH3T3 cells with the adenovirus for over-expression of PTPMeg2. Cells were suspended in 1 ml physiological saline for preparation of injection into mice. BALB/c-nu/nu mice at 5 weeks of age were subjected to bilateral subcutaneous injections with 1.0 × 10^7 ^(MCF-7) or 5.0 × 10^6 ^(MDA-MB-231) or 5.0 × 10^5 ^(v-Src/NIH3T3) cells in a volume of 0.1 ml saline. Tumor volume defined as (length × width^2^)/2 was measured every two days with a caliper up to study termination. Tumor growth curves were drawn according to the average of tumor volumes (mm^3^). All animal experiments were performed in accordance with the institutional animal experiment guidelines.

### Patient samples and immunohistochemistry

The formalin-embedded tissue samples from 73 patients with breast carcinomas diagnosed between 2008 and 2010 were obtained from the Surgical Pathology in the TangShan People's Hospital. All breast cancer specimens from female patients were obtained from clinical surgery. Information of age, histological type, differentiation grade, and lymph node metastasis of breast carcinomas were obtained from the Surgical Pathology Files in the hospital. The clinicopathological diagnosis on the tumor status was evaluated by the clinical pathologists in the hospital. All samples used in the study were approved by the TangShan People's Hospital Ethical Committee under the guidance of tissue collection procedure with informed consent.

Sections of formalin-fixed breast carcinoma tissues were treated with 0.3% hydrogen peroxidase/methanol and incubated with primary antibodies followed by incubation with secondary antibodies (biotin-labeled; Santa Cruz) and third antibodies (peroxidase-labeled; Santa Cruz). Samples were developed using DAB as substrates (Santa Cruz). Scoring criteria for tumor degrees as reported previously were used [28]. Briefly, the grade was classified as 0 for negative, 1 for weak (< 10%), 2 for moderate (10-25%), 3 for strong (26-75%) and 4 for very strong (> 75%) staining according to percentage of positively staining cells. The staining index was subsequently obtained by multiplication of the proportion and intensity and calculated index was finally assessed by a simplified score (score 0, index 0-1; score 1, index 2-4; score 2, index 6-8; score 3, index 9-12). Samples with staining score of at least 1 were classified as positive staining, score 2 and 3 were strong positive staining. The percentage of pSTAT3 nuclear positive cells were used to classify the grade of its expression as negative (< 5%), weak (6-50%), and strong (51-100%).

### Statistical analysis

All experiments were repeated at least three times. The Student's *t *test was used to evaluate the significance of differences between experimental and control groups. Data were analyzed by one-way ANOVA with SPSS13.0 (SPSS, Int, Chicago, IL). Frequencies of PTPMeg2, STAT3 and pSTAT3 expressions among cancer samples were analyzed by the *x^2 ^*test with a modification by the Fisher's exact test to account for frequency values < 5. The correlation between protein levels was evaluated by the pair-wise Pearson correlation coefficient and by bi-dimensional hierarchical clustering. All *P*s reported were two-sided. Significance was defined at the level of *P ≤ *0.05.

## Results

### PTPMeg2 interacts with STAT3 in mammalian cells

To search for negative regulators of STAT3, we examined the possibility of its interaction with different phosphatases, and PTPMeg2 was identified as a potential interacting protein. To confirm the interaction, Myc-PTPMeg2 and Flag-STAT3 were co-expressed in HEK 293T cells and co-immunoprecipitation and GST pull-down experiments were performed. The results showed that PTPMeg2 interacts with STAT3 *in vitro *(Figure 1A and 1B). Interestingly, we observed that PTPMeg2 preferentially interacted with STAT3 as it had either a weak or no interaction with STAT5 or STAT1 (Figure 1C). An *in vivo *interaction of endogenous PTPMeg2 and STAT3 proteins was observed in the mouse brain tissue (Figure 1D, left panel) and breast cancer MCF7 cells (Figure 1D, right panel). All these results suggested that PTPMeg2 interacts with STAT3 under physiological and pathological conditions.

**Figure 1:** **PTPMeg2 interacts with STAT3**. (A) PTPMeg2 was co-immunoprecipitated with STAT3 in mammalian cells. Lysates prepared from HEK293T cells expressing Flag-STAT3 and Myc-PTPMeg2 were precipitated with an anti-Flag antibody and the precipitants were blotted by an anti-Myc antibody. (B) STAT3 interacts with PTPMeg2 physically *in vitro*. GST or GST-STAT3 fusion proteins were mixed with the Myc-PTPMeg2 prepared from cells (C) PTPMeg2 preferentially interacts with STAT3. Myc-PTPMeg2 was co-expressed with Flag-tagged STAT3 (S3), STAT1 (S1) or STAT5a (S5a) in 293T cells. (D) PTPMeg2 interacts with STAT3 *in vivo*. Lysates from the mouse brain tissue and breast cancer MCF7 cells were used in co-immunoprecipitation assays to demonstrate the endogenous protein interaction with an anti-STAT3 antibody (C20) and anti-PTPMeg2 rabbit polyclonal antibody. (E) PTPMeg2 interacts with phosphorylated STAT3. A reciprocal immunoprecipitation assay was performed with an anti-Myc antibody or an anti-Flag antibody for the lysates of HEK293T cells under IL-6 stimulation for 30 min. (F) IL-6 induces the interaction of STAT3 and PTPMeg2 *in vivo*. An immunoprecipitation assay was performed using the endogenous proteins in MCF7 cells stimulated by IL-6 for 30 min. (G) PTPMeg2 decreases the accumulation of pSTAT3 in the nucleus. MCF7 cells transfected with STAT3 and/or PTPMeg2 WT/CS were treated without or with IL-6 for 30 min. Cells were immunostained with an anti-PTPMeg2 (FITC) and an anti-Flag antibody (TRITC, for Flag-STAT3). DAPI was used for nuclear staining. Scale, 10 μm.

### PTPMeg2 interacts with both phosphorylated and unphosphorylated forms of STAT3

To determine if the interaction of PTPMeg2 with STAT3 is regulated by cytokines, HEK 293T cells transfected with Flag-STAT3 and Myc-PTPMeg2 were stimulated by IL-6 for 30 min. A reciprocal immunoprecipitation experiment indicated that the interaction of PTPMeg2 and STAT3 was increased dramatically under stimulation of IL-6 (Figure 1E). Interestingly, we observed a strong band of phosphorylated STAT3 in a complex precipitated with an anti-Myc antibody (for Myc-PTPMEG2) (Figure 1E). Consistently we observed that IL-6 induced the interaction of endogenous STAT3 and PTPMeg2 in MCF7 cells (Figure 1F). These results suggest that PTPMeg2 interacts with the phosphorylated form of STAT3 (pSTAT3). Based on the observation that PTPMeg2 interacts with STAT3 in the absence of IL-6, we concluded that PTPMeg2 interacts with both the phosphorylated and unphosphorylated STAT3.

To reveal the cellular location of the PTPMeg2/STAT3 complex, we performed an immunofluorescence staining assay in MCF7 cells transfected with STAT3 and PTPMeg2. The results showed that STAT3 was located in the cytoplasm under a quiet condition, but translocated into the nucleus after IL-6 stimulation (Figure 1G, b2-b3). When STAT3 was co-expressed together with PTPMeg2, a notable co-localization of the two proteins in the cytoplasm was observed (Figure 1G, c3). Interestingly, we observed that STAT3 remained in the cytoplasm under the stimulation of IL-6 when PTPMeg2 was co-expressed (Figure 1, 2, 3). This result suggests that PTPMeg2 blocks the translocation of STAT3 from the cytoplasm into the nucleus upon IL-6 stimulation. To support this notation, a mutant PTPMeg2CS, which lost the ability to dephosphorylate STAT3, failed to block STAT3 localization into the nucleus in response to IL-6 stimulation (Figure 1, 2, 3). These results suggest that STAT3 colocalizes with PTPMeg2 in the cytoplasm and overexpression of PTPMeg2 inhibits the translocation of STAT3 upon cytokine stimulation.

**Figure 2:** **PTPMeg2 enhances dephosphorylation of STAT3**. (A) PTPMeg2 decreases the level of pSTAT3. Levels of pSTAT3(Tyr705) were examined in the HEK293T cells transfected with Flag-STAT3 and different forms of PTPMeg2 in the presence or absence of IL-6 (10 ng/ml) for 30 min. (B) PTPMeg2 increases the dephosphorylation of STAT3. HEK293T cells were treated with IL-6 (10 ng/ml) for 30 min, followed by a starvation (shown as withdrawal) for different times. (C) PTPMeg2 promotes the STAT3 dephosphorylation rate. HEK293T cells were treated with IL-6 (10 ng/ml) for 30 min, followed by starvation for different times. The dynamic changes of the pSTAT3 (Tyr705) levels demonstrates the dephosphorylation rate of STAT3. (D) PTPMeg2 mediates STAT3 dephosphorylation in a dose dependent manner. HEK293T cells were transfected with Flag-STAT3 (2 μg/well) and different amounts of PTPMeg2 in a 6 well plate. (E) PTPMeg2 dephosphorylates STAT3 *in vitro*. Different amounts of purified GST-PTPMeg2 (10, 5 and 2.5 μg/tube) was added to purified pSTAT3 in a PTPase buffer at 37°C for 30 min. pSTAT3 was prepared in HEK293T cells transfected with Flag-STAT3 for 48 h and then stimulated with IL-6 for 30 min. (F) The PTP domain of PTPMeg2 contributes to STAT3 dephosphorylation. Myc-PTP domain, Myc-SEC domain and different deletions of PTPMeg2 were co-transfected with Flag-STAT3 for 48 h before stimulation with 10 ng/ml IL-6 for 30 min.

**Figure 3:** **PTPMeg2 decreases the transcription activity of STAT3**. (A) PTPMeg2 inhibits IL-6-stimulated STAT3 transcriptional activity. Luciferase assays were performed using MCF7 cells with transient expression of Myc-PTPMeg2 and Flag-STAT3, transfected with APRE-Luc reporter and pRL-TK (as an internal control). Relative luciferase activities were normalized with the internal control. Results are presented as mean ± SD from three independent experiments. (B) PTPMeg2 inhibits STAT3-mediated transcriptional activity in a dose dependent manner. Different amounts of PTPMeg2 were co-expressed with STAT3 in the presence or absence of IL-6 stimulation. Different amounts of PTPMeg2CS were also co-expressed with STAT3. (C) The PTP domain of PTPMeg2 inhibits the STAT3 transcriptional activity. Different domains and deletions of PTPMeg2 were co-expressed with Flag-STAT3 in the MCF7 cells and luciferase assays were performed as above. (D) Depletion of PTPMeg2 results in an enhanced STAT3 transcriptional activity. An shRNA targeting PTPMeg2 was co-expressed with STAT3 in MCF7 cells transfected with APRE-Luc reporter and pRL-TK under stimulation of IL-6. Luciferase activities were assayed as above. (E) Levels of pSTAT3(Tyr705) and STAT3 were examined in the MCF7 cells overexpressed and depleted PTPMeg2 in separated membranes from the same lysates. (F) PTPMeg2 has no effect on the STAT1 transcriptional activity. M67 luciferase reporters were co-transfected into MCF7 cells with STAT1 and PTPMeg2, in the presence or absence of IFN-gamma. Luciferase activities shown are mean ± SD of three independent experiments.

### PTPMeg2 enhances dephosphorylation of STAT3

Our observation that over-expression of PTPMeg2 blocks STAT3 translocation implied that PTPMeg2 may regulate STAT3 phosphorylation. Since PTPMeg2 is a phosphatase, we determined to examine whether PTPMeg2 dephosphorylates STAT3. To this end, HEK293T cells were transfected with Flag-STAT3 and Myc-PTPMeg2 plasmids under IL-6 treatment for 30 min. The results showed that the level of pSTAT3 was decreased when PTPMeg2 was co-expressed with STAT3 (Figure 2A). In contrast, transfection of mutant PTPMeg2CS failed to decrease the level of pSTAT3 (Figure 2A). To examine whether the decreased level of pSTAT3 is induced by a dephosphorylation or protein degradation process, the level of pSTAT3 was examined after withdrawal of IL-6 and in the presence of MG132, an inhibitor of proteosome. Results showed that the level of pSTAT3 was decreased much more quickly when PTPMeg2 was over-expressed than that without PTPMeg2 (Figure 2B). At the same time, the level of pSTAT3 remained unchanged in the presence or absence of MG132 (Figure 2B). These dada indicated that PTPMeg2 induces dephosphorylation of pSTAT3 rather than its degradation. Furthermore, we showed that over-expression of PTPMeg2 promoted the dephosphorylation of STAT3 at the residue Tyr 705 but had no effect on the phosphorylation level of pSTAT3 at the residue Ser727 (Figure 2C). The role of PTPMeg2 on the dephosphorylation of pSTAT3 (Tyr705) was further confirmed in a dosage dependent experiment (Figure 2D). These results suggested that ectopic expression of PTPMeg2 regulates the tyrosine phosphorylation of STAT3.

To further confirm the role of PTPMeg2 on dephosphorylation of STAT3, purified GST-PTPMeg2 and GST-PTPMeg2CS fusion proteins were used to incubate with pSTAT3 prepared from mammalian cells for an *in vitro *phosphatase activity experiment. The results showed that the tyrosine phosphorylation level of STAT3 was dramatically reduced when GST-Meg2 protein was added in a dose dependent manner (Figure 2E). As controls, addition of GST or GST-PTPMeg2CS had no effect on the level of pSTAT3 (Figure 2E, lane 1 to 2). This result indicated that STAT3 is a substrate of PTPMeg2. To address whether the PTP domain of PTPMeg2 has the phosphatase activity, the SEC domain, PTP domain and mutations of different deletions (ΔSEC, ΔPTP) were generated to examine the effect on the level of pSTAT3. A Western blot result showed that both PTP domain and ΔSEC domain had the ability to dephosphorylate pSTAT3 (Figure 2F, lanes 4 and 5). These data indicated that the PTP domain is responsible for the phosphatase activity of PTPMeg2, which is in consistency with the role of the PTP domain in other phosphatases.

### PTPMeg2 suppresses the transcriptional activation of STAT3

We questioned whether PTPMeg2 regulates the transcriptional activity of STAT3 based on its interaction with STAT3. To this end, we used an APRE luciferase reporter, which responds to STAT3 activation, to examine the effect of PTPMeg2 on STAT3 mediated transcriptional activity. The results showed that over-expression of PTPMeg2 in MCF7 cells resulted in a decrease of the luciferase activity in response to over-expressed STAT3 and stimulation of IL-6 (Figure 3A). The inhibitory role of PTPMeg2 on the STAT3-mediated luciferase activity was dose dependent (Figure 3B, left columns). Interestingly, when the mutant PTPMeg2CS was increasingly expressed the STAT3-mediated luciferase activity was increased (Figure 3B, right columns). These results suggest that the mutant PTPMeg2CS acts as a dominant negative antagonist of endogenous PTPMeg2 in regulating STAT3 phosphorylation. In consistence, depletion of the PTP domain impaired the activity of the phosphatase (Figure 3C). Finally, we showed that depletion of PTPMeg2 by three shRNAs increased the luciferase activity mediated by STAT3 (Figure 3D) while these shRNAs dramatically recovered the phosphorylation of the endogenous STAT3 protein (Figure 3E). In contrast, over-expression of PTPMeg2 had no effect on the transcriptional activity of STAT1 in response to INF-gamma stimulation (Figure 3F). These results indicate that PTPMeg2 inhibits STAT3 activation with certain specificity.

### PTPMeg2 inhibits breast cancer cell proliferation and tumor growth in nude mice

Since STAT3 phosphorylation is highly related to tumorigenesis, we attempted to examine whether PTPMeg2 could affect tumor progression. For this purpose, we used two human breast cancer cell lines MCF7 and MDA-MB-231. We observed that the endogenous PTPMeg2 protein level was low in MDA-MB-231 cells but high in MCF7 cells while the level of endogenous pSTAT3 displayed a reversed trend (Figure 4A). Therefore we determined to establish a gain-of-function model in MDA-MB-231 cells and a loss-of-function model in MCF7 cells.

**Figure 4:** **PTPMeg2 inhibits breast cancer cell proliferation and tumor growth in nude mice**. (A) PTPMeg2 expression correlates with the pSTAT3 level in breast cancer cells. The levels of pSTAT3, STAT3 and PTPMeg2 are shown. (B) Depletion of PTPMeg2 results in an increased level of pSTAT3 and expression of downstream gene expression. An shRNA targeting PTPMeg2 was stably expressed in MCF7 cells (MCF7/shPTPMeg2). Two downstream proteins CyclinD1 and Bcl-xL were examined. (C) Silencing PTPMeg2 increases the MCF7 cell proliferation. MCF7 stable cell lines were examined by an MTT assay. (D-F) Depletion of PTPMeg2 increases growth of tumors from MCF7 cells in nude mice. 1 × 10^7 ^MCF7 cells stably expressing shPTPMeg2 were injected s.c. into the right flanks of 6-week-old female nude mice (n = 6). Tumor weights (D), xenograft tumors (E), tumor sizes (F) are shown. (G) Over-expression of PTPMeg2 inhibits pSTAT3 and expression of its targeted genes. MDA-MB-231 cells were infected with Ad/PTPMeg2 or Ad/GFP. (H) Over-expression of PTPMeg2 inhibits MDA-MB-231 cell proliferation. MDA-MB-231 cells were examined by an MTT assay. (I-K) Over-expression of PTPMeg2 represses tumor growth. Tumor formation was observed in nude mice injected with 2 × 10^6 ^MDA-MB-231cells infected with Ad/PTPMeg2 or Ad/GFP. Xenograft tumors (I), tumor weights (J) and tumor volumes (K) are shown. All the data were obtained from 6 Balb/c-nu nude mice. Tumor formation was examined in nude mice injected with 6 × 10^6 ^MDA-MB-231cells infected with pMSCV/PTPMeg2 or pMSCV/vector virus. Xenograft tumors (L), tumor weights (M) and tumor volumes (N) are shown.

To address the increased pSTAT3 was the cause of decreased PTPMeg2, we stably depleted PTPMeg2 by using an shRNA targeting PTPMeg2 in MCF7 cells. A Western blot analysis showed that pSTAT3 was dramatically increased when PTPMeg2 was depleted (Figure 4B, right lane). Intriguingly, a cell proliferation experiment result showed that the growth of MCF7 cells was increased when PTPMeg2 was depleted (Figure 4C). An *in vivo *tumor growth experiment in a xenograft tumor model in mice showed that MCF7 cells with stable depletion of PTPMeg2 formed larger tumors than mock transfected cells (Figure 4D-E) and grew more rapidly (Figure 4F). On the other hand, we over-expressed PTPMeg2 in MDA-MB-231 cells using an adenovirus expression system. The results showed that MDA-MB-231 cells infected with the adenovirus expressing PTPMeg2 had a lower level of endogenous pSTAT3 than the cells infected with a control adenovirus (GFP) (Figure 4G, right lanes). And these cells grew much more slowly (Figure 4H) and the cells formed smaller sized tumors (Figure 4I-J) and had slower tumor growth rate (Figure 4K), lower tumor weight (Figure 4J) and slower tumor growth (Figure 4K). To further confirm the inhibitory role of PTPMeg2 on tumor growth in a moderate expression system, we used the retroviral system to ectopically express PTPMeg2 (pMSCV/PTPMeg2) in MDA-MB-231 cells. The results were similar to that using the adenovirus expression system (Figure 4L-N). All these results indicated that PTPMeg2 inhibits STAT3 phosphorylation directly and PTPMeg2 is a tumor suppressor.

To confirm the inhibitory role of PTPMeg2 on tumor growth is depended on regulation of STAT3 phosphorylation, we used v-Src transformed NIH3T3 fibroblasts in a xenograft tumor model. The result showed that v-Src transformed cells had a much higher STAT3 phosphorylation level than non-transformed cells and over-expression of PTPMeg2 significantly decreased the level of pSTAT3 (Figure 5A). Consistent with the decreased level of pSTAT3, the tumor size (Figure 5B), weight (Figure 5C) and tumor growth (Figure 5D) from v-Src transformed cells were decreased when PTPMeg2 was forcedly expressed. These data implied a correlation of PTPMeg2-reduced tumor growth and the decreased level of pSTAT3. To address whether pSTAT3 is a key target by PTPMeg2, we examined the cell proliferation ability in the STAT3 KO cells. A MTT experiment indicated that overexpression of PTPMeg2 inhibited the cell growth dramatically in wild-type cell but had no effect in the STAT3 KO cells (Figure 5E-F), suggesting that the inhibitory role of PTPMeg2 on the cell proliferation is depended on STAT3. Together with the biochemical data, these results suggested that the ability of PTPMeg2 to inhibit the tumor growth and cell proliferation is depending on its role of regulation of phosphorylated STAT3.

**Figure 5:** **The correlation of the PTPMeg2 expression and the pSTAT3 level**. (A-D) Over-expression of PTPMeg2 decreases the tumor growth of v-Src transformed fibroblasts. (A) v-Src activated pSTAT3 was decreased by Ad/PTPMeg2. A Western blot was used to show the indicated proteins. STAT3 and pSTAT3 were examined in separated membranes from the same lysates. (B-D) 5 × 10^5 ^v-Src/NIH3T3 cells infected with Ad/PTPMeg2 or Ad/GFP were used to inject s.c. into the right (Ad/PTPMeg2) and left (Ad/GFP) flanks of 6-week-old male nude mice (n = 5). Xenograft tumors (B), tumor weights (C) and tumor volumes (D) are shown. (E) Over-expression of PTPMeg2 decreases the STAT3^+/+ ^cell proliferation. Mouse hepatic STAT3^+/+ ^and STAT3^+/+^cells infected with the indicated adenovirus were used to examine the proliferation rate by an MTT assay. Results were averaged from three repeats. (F) A Western blot was used to show the indicated proteins. (G) A high level of pSTAT3 is correlated with a low expression of PTPMeg2 in the breast carcinoma. Representative images of immunohistochemical staining of PTPMeg2, pSTAT3 and STAT3 are shown. All the tumor tissues were derived from surgery sections. Peri-tumor (P) or tumor (T) tissues are marked with dotted lines. Scale bars, 50 μm.

In consistence with the tumor growth experiment, we examined the expression of STAT3 downstream genes. The result showed that both Bcl-xL and cyclin D1 were dramatically increased when PTPMeg2 was depleted in MCF7 cells (Figure 4B). In contact, Bcl-xL and cyclin D1 were decreased when PTPMeg2 was over-expressed in MDA-MB-231 cells (Figure 4G). We observed no alteration of STAT3 expression but the phosphorylated STAT3 level was changed with either over-expression or depletion of PTPMeg2 (Figure 4B, G). These results suggest that PTPMeg2 regulates STAT3 phosphorylation and thereafter the downstream gene expression.

To address whether PTPMeg2 regulates STAT3 dephosphorylation in human tumors, we examined the correlation of pSTAT3 level and expression of PTPMeg2 in human breast cancers. The result showed that expression of PTPMeg2 was in a strong positive status in peritumoral tissues (90% = 37/41) and in a negative status in paired tumor tissues (83% = 59/71) (Figure 5E, Table 1). In contrast, pSTAT3 remained at a low (or negative) level in the peritumoral tissues but at a high level (71% = 52/73) in the paired tumor tissues (Figure 5E). We observed a negative correlation between PTPMeg2 expression and the pSTAT3 level (spearman's correlation coefficient was -3.33, *p *= 0.004, Table 2) from a Spearman's correlation test. The analysis also revealed that the increased STAT3 level was correlated with reduced PTPMeg2 expression in the breast carcinoma (correlation coefficient is -2.65, *p *= 0.023, Table 2). These data indicated that PTPMeg2 might be an important regulator of STAT3 dephosphorylation in tumors.

**Table 1:** The expression level of PTPMeg2 in the breast cancer samples

	PTPMeg2 positive	PTPMeg2 negative	Total
Tumor	14	59	73
Peri-tumor	37	4	41
total	51	63	114

*X*^2 ^= 53.262, *p *= 0.000

**Table 2:** Correlation of pSTAT3 with PTPMeg2 expression in breast cancer

		PTPMeg2				
				
	number	negative	weak	strong	correlation coefficient	P*
pSTAT3	73				r = - 3.33**	0.004
negative	12	6	5	1		
Weak	9	7	1	1		
strong	52	46	5	1		
STAT3	73				r = - 2.65*	0.023
negative	4	1	3	0		
Weak	4	3	1	0		
strong	65	55	7	3		
ER	60				r = 0.280	0.834
negative	23	20	3	0		
Weak	11	9	2	0		
strong	26	22	4	0		
PR	60				r = 0.212	0.105
negative	25	23	2	0		
Weak	19	14	2	0		
strong	14	14	5	0		
Her2	70				r = - 1.53	0.203
negative	25	20	5	0		
Weak	10	9	1	1		
strong	35	32	3	0		

r* < 0.05, r** < 0.01.

## Discussion

Targeting pSTAT3 has becoming an important strategy for cancer therapies [29] since hyper-phosphorylation of STAT3 at tyrosine residues is associated with various types of human cancers including breast cancer. The hyper-phosphorylated STAT3 was caused by either the over-activation of tyrosine kinases or the impaired function of tyrosine phosphatases. While many kinases have been reported to activate STAT3 in tumors, it is still interesting to identify a direct STAT3 phosphatase. In this study, we found that PTPMeg2 is a strong phosphatase directly interacting with STAT3 and mediating STAT3 dephosphorylation.

We have presented several lines of evidence demonstrating STAT3 is a substrate of PTPMeg2. First, PTPMeg2 physically and pathologically interacts with STAT3. Significantly, PTPMeg2 exhibits a strong affinity for pSTAT3 and STAT3. Next, PTPMeg2 dephosphorylated pSTAT3 in time- and dose-dependent manners. Third, the catalytically inactive mutant of PTPMeg2 lost the negative role in pSTAT3. Fourth, deletion of the lipid-binding domain of PTPMeg2 has no effect on the dephosphorylation. On the contrary, depleting PTPMeg2 enhances the level of pSTAT3 in cells and results in the cell proliferation and tumor growth in nude mice. Consistent with the biochemistry and cellular biology data, we observed that the negative correlation between the expression of PTPMeg2 and pSTAT3 in human breast cancer samples. All the results are consistent and intercomparable in demonstrating the role of PTPMeg2 in regulation of STAT3 activity in the breast cancer. However, we can not exclude the possibility that PTPMeg2 may target other substance. In this study, we demonstrated that the inhibitory role of PTPMeg2 on tumor growth was mainly through dephosphorylation of STAT3.

Previous studies reported that several PTPs such as PTPN1, PTPN3, and PTPN6 [30] have oncogenic properties but other PTPs including PTPN12 [31] have tumor suppressor features. In this study, we found that PTPMeg2 is a tumor repressor preferentially dephosphorylating STAT3. We have used several cell models to demonstrate that enforced expression of PTPMeg2 inhibited tumor cell growth and depletion of PTPMeg2 resulted in enlarged tumors. Intriguingly we found that the expression of PTPMeg2 was negative in human breast cancer while it remained high in the peritumoral tissues. This expression pattern is similar to that of PTPN7 [32] and PTPN13 [33], which were reported to be at a global loss in a wide range of cancers including breast, kidney, and esophageal cancers. Recently, PTPN13 was reported to loss its activity through somatic mutations, allelic loss, or promoter methylation in some tumors [34]. Whether PTPMeg2 has such a kind of mutations in tumors remains unclear.

It has reported that PTPL1/PTPN13 regulated breast cancer cell aggressiveness through a direct inactivation of Src kinase [33] and PTPN12 inhibits breast cancer metastasis through multiple targets including EGFR1, Her2 and Src kinase [31]. A previous study reported that PTPMeg2 targets EGFR and Her2 [20]. In this study, we found that PTPMeg2 directly interacts with STAT3. Interestingly, when we used v-Src to activate STAT3 phosphorylation, we observed that PTPMeg2 strongly mediated dephosphorylation of STAT3 (Figure 5). However, we did not observe any interaction of v-Src with PTPMeg2. This result implies that PTPMeg2 directly targets STAT3 activated by v-Src. Since STAT3 associates with EGFR or Her2, it is possible that PTPMeg2 interacts with the STAT3/EGFR complex, as observed by a previous study [20]. Whether the interaction of PTPMeg2 with STAT3 requires other partners will be an interesting question in future studies.

Another interesting observation is that PTPMeg2 mediates dephosphorylation of STAT3 at residue Try705 while is has no effect of the phosphorylation of STAT3 at residue Ser727. This seems reasonable since PTPMeg2 is in the family of protein tyrosine phosphatases. We predict that the dephosphorylation of STAT3 at other non tyrosine residues is likely mediated by other phosphatases to be further identified.

## Conclusion

In summery, we demonstrated that the cytoplasmic phosphatase PTPMeg2 directly mediates the dephosphorylation of pSTAT3 and negatively regulates STAT3 activity. Down regulated expression of PTPMeg2 is correlated with elevated phosphorylated STAT3 in human breast cancer tissues. Recovery of PTPMeg2 by adenovirus/retrovirus results in tumor regression in nude mouse models.

## Abbreviations

EGFR: Epidermal growth factor receptor; GST: Glutathione S-transferase; IL-6: Interleukin-6; INF: Interferon; JAK: Janus Associated Kinase; KO: Knockout; PTP: Protein Tyrosine Phosphatase; PTPMeg2: Protein Tyrosine Phosphatase Meg2; SOCS 3: Suppressor of Cytokine Signaling 3; STAT: Signal Transducers and Activators of Transcription; v-Src: viral-sarcoma; shRNA: short hairpin RNA; WT: Wild Type.

## Competing interests

The authors declare that they have no competing interests.

## Authors' contributions

FS: IHC, IP, mouse experiments and draft manuscript writing; FR: IP, IF experiments and statistical analysis; YR: construction of the plasmids and IP experiments; YW: luciferase experiments; YG: mouse experiments; YW: IF experiments; MF: cell culture and IHC experiment; YJ: pathology analysis; YL: experiment design and discussion; ZJZ: experiment design and discussion; KM: experiment design and discussion; ZC: experiment design and direction, manuscript writing. All authors read and approved the final manuscript.

## Authors' information

Mengyao Feng is currently a student in Sun Yat-Sen University in China. Kun Meng is currently at Suite A205, 5 Shangdi Kaituo Rd., Haidian, Beijing, 100085, China.
